The article "A candidate Chinese medicine preparation-Fructus Viticis Total Flavonoids inhibits stem-like characteristics of lung cancer stem-like cells" was retracted in 2022. Reasons: manipulated images; duplicated images; signs of a paper mill.

# A candidate Chinese medicine preparation-Fructus Viticis Total Flavonoids inhibits stem-like characteristics of lung cancer stem-like cells

**DOI:** 10.1186/s12906-016-1341-4

**Published:** 2016-09-15

**Authors:** Xiaocheng Cao, Hui Zou, Jianguo Cao, Yinghong Cui, Shuwen Sun, Kaiqun Ren, Zhenwei Song, Duo Li, Meifang Quan

**Affiliations:** 1 College of Life Science, Hunan Normal University, Changsha, China; 2 Laboratory of Medicine Engineering, College of Medicine, Hunan Normal University, Changsha, China

**Keywords:** Lung cancer, Cancer stem cell, Fructus Viticis Total Flavonoids, AKT, Therapeutic action

## Abstract

**Background:**

Cancer stem cells (CSCs) are considered as the origin of tumor relapse. Here, we investigated the effects of Fructus Viticis total flavonoids (FVTF) on the characteristics of lung cancer stem-like cells (LCSLCs) derived from human small cell lung cancer NCI-H446 cell line and its potential mechanism.

**Methods:**

Human small cell lung cancer NCI-H446 cell line was cultured in vitro. The CD133^+^ cells were sorted from NCI-H446 cell line by magnetic separation.

The suspended culture with stem cell-conditioned medium was used to amplify CD133^+^ sphere-forming cells (SFCs). The stem cell characteristics of CD133^+^ SFCs were evaluated using cell self-renewal capacity by tumor sphere formation assay, migration and invasion capacity by Transwell assay, tumorigenicity by xenograft model in nude mouse and cancer stem cell markers expression levels by western blot. The effects of FVTF on the properties of LCSLCs were examined by tumorsphere formation assay and transwell chamber assay. The expression level of p-Akt was determined by western blot analysis.

**Result:**

CD133^+^ SFCs derived from human small cell lung cancer NCI-H446 cells exhibited stemness properties of tumorsphere formation and tumorigenesis capacity comparing to the parental cells. FVTF relative selectively inhibited the proliferation of LCSLCs, suppressed tumor sphere forming capacity and migration and invasion of LCSLCs, and down-regulated the protein expression of stem cell markers (CD133, CD44 and ALDH1), self-renewal associated transcription factors (Bmi1, Nanog and OCT4) and invasion associated transcription factors (Twist1 and Snail1) in a dose-dependent manner. Moreover, we found that FVTF treatment could significantly decrease the phosphorylation level of Akt in LCSLCs. Meanwhile, LY294002 and FVTF synergistically inhibited the characteristics of LCSLCs.

**Conclusion:**

FVTF inhibits the characteristics of LCSLCs through down-regulating expression of p-Akt.

## Background

Lung cancer is one of the most common malignancies worldwide and it ranks as the most frequent cause of cancer-related deaths especially in urban areas of China [1, 2]. The most common subtypes of lung cancer are non-small cell lung cancer (NSCLC) and small cell lung cancer (SCLC). And the latter is the most aggressive form of lung cancer, with a high invasive capacity and greater tendency for development of early metastasis [3]. Despite all kinds of conventional therapeutic regime applied in clinical treatment, lung cancer has a dismal 5-year survival rate due to failure of currently available therapeutic approaches and finally resulting in disease relapse [4].

The article "A candidate Chinese medicine preparation-Fructus Viticis Total Flavonoids inhibits stem-like characteristics of lung cancer stem-like cells" was retracted in 2022. Reasons: manipulated images; duplicated images; signs of a paper mill.

Researchers frequently attributes the therapy resistance of lung cancer to cancer stem cells(CSCs) within the tumors. Increasing evidence has indicated that many types of solid cancer, including lung cancer, are originated from and maintained by a minor subpopulation of CSCs [5, 6]. These cells possess the capacity of continuous self-renewal, differentiation and initiating tumor formation as well as show increased resistance to radiation and chemotherapy. CSCs are considered as the origin of tumor relapse.

Recently, various methods based on specific cell surface markers, the capacity of cells to exclude membrane permeable dyes or the ability of tumor sphere formation for single cell in suspension in serum-free medium have been used for CSCs isolation and characterization [7–9]. Similar to other solid tumors, several putative surface markers for lung CSC(LCSCs) have been identified, including CD133 and CD44 [6, 10–12]. Eramo et al. found the existence of a rare population of undifferentiated cells expressing CD133 in small cell and non-small cell lung cancer for the first time. These minor population of CD133+ tumorigenic cells able to self-renew and give rise to an unlimited progeny of differentiated tumor cells are named lung cancer stem cells (LCSCs) [10]. However, another study by Meng et al. found out that both the CD133+ and CD133- subpopulations from SCLC cells contain similar numbers of cancer stem cells, which suggest that CD133 alone cannot be used as a stem cell marker for the SCLC [7]. In addition, Jiang et al. also demonstrated that Aldehyde dehydrogenase 1 (ALDH1) is a tumor stem cell-associated marker in lung cancer [8]. Taken together, although no certain specific cell markers for LCSCs have been defined yet, we think that the suspended culture with stem cell-conditioned medium can be at least used as a crucial approach for enrichment of LCSCs. Therefore, developing new chemotherapy agents that can target these LCSCs has profound implications for cancer chemoprevention and therapy.

Fructus Viticis (Manjingzi is the Chinese name), the dried ripe fruit of Vitex trifolia L. (family Verbenaceae), is a traditional Chinese medicine possessing a broad range of pharmacological activities [13–15]. Fructus Viticis contains large amounts of flavonoids, including casticin, luteolin, apigenin, isoorientin, hesperidin, isovitexin and so on [16–18]. Accumulating studies have substantiated the anti-tumor properties of these flavonoids in a diverse range of human cancer cells and their xenograft models in mice [19, 20]. FVTF(Fructus Viticis Total Flavonoids), an independent innovation of our laboratory, is a candidate Chinese medicine preparation extracted from Fructus Viticis (National invention application No. ZL 201210591146.9).

The article "A candidate Chinese medicine preparation-Fructus Viticis Total Flavonoids inhibits stem-like characteristics of lung cancer stem-like cells" was retracted in 2022. Reasons: manipulated images; duplicated images; signs of a paper mill.

In the present study, we obtained the CD133^+^ sphere-forming cells (SFCs) from NCI-H446 cells by employing CD133^+^ magnetic separation and stem cell-conditioned medium culture method. Furthermore, we confirmed the LCSLCs characteristic of SFCs by compared the self-renewal capacity, stem cell markers expression levels, and tumorigenicity of SFCs and non-sorting cells, namely parental cells. The aims of this study were to investigate whether FVTF could inhibit the characteristics of LCSLCs and the potential mechanisms involved.

## Methods

### Drugs and reagents

The Fructus Vititcis was purchased from Yuling Zhonggui Pharmaceutical Company (Yuling, Guangxi province, China). Prof. Bing-Qing Zhao (Department of Pharmacy, Medical College of Hunan Normal University) identified the specimens. A voucher specimen has been deposited in the Department of Pharmacy, Medical College of Hunan Normal University (No. MJZ-001). Fructus Viticis Total Flavonoids(FVTF) was extracted and prepared from Fructus Viticis according to the patent specification (National invention application of China No. ZL 201210591146.9), present as brown powder. The measured amounts of total flavonoids in drying FVTF were 53 % calculated based on rutin.

DMEM medium(High glucose), DMEM/F12 medium, fetal bovine serum, 0.25 % trypsin(containing EDTA) and phosphate buffered saline (PBS) were purchased from Hyclone(Logan, UT, USA). Recombination human fibroblast growth factor (bFGF), epidermal growth factor (EGF) and B27 were purchased from eBioscience. Hematoxylin and Eosin Staining Kit, Matrigel (BD Biosciences, USA). Cell lysis buffer, trypan Blue, penicillin and streptomycin (Invitrogen Life Technologies) and bovine serum albumin were purchased from Hunan Clonetimes Biotech Co., Ltd. (Changsha, Hunan). Human insulin were purchased from Beijing Dingguo Changsheng Biotechnology Co. Ltd. Mouse monoclonal antibodies anti-CD44, ALDH1, Bmi1, Nanog, Oct4, Twist, Snail, p-Akt (Ser473), Akt, β-actin were from Cell Signaling Technology (Beverly, MA, USA).

The article "A candidate Chinese medicine preparation-Fructus Viticis Total Flavonoids inhibits stem-like characteristics of lung cancer stem-like cells" was retracted in 2022. Reasons: manipulated images; duplicated images; signs of a paper mill.

### Cell culture

Human small cell lung cancer (SCLC) cell line NCI-H446 was purchased from Keygen biotechnology Co., Ltd. (NanJing, China), and was maintained in DMEM (High glucose) supplemented with 10 % fetal bovine serum, 100 U/mL penicillin and 100 μg/mL streptomycin in an incubator containing 5 % CO_2_ at 37 °C.

### Magnetic separation of CD133^+^ cells

The CD133^+^ positive cells were sorted from NCI-H446 cell line using magnetic separation (Miltenyi Biotec, Germany) according to the manufacturer’s instruction. Briefly, a single-cell suspension was firstly prepared and the cell number were determined before magnetic labeling. Cells were collected by centrifuge at at 300 × g for 10 min and the cell pellet were resuspended in 60 μL of buffer per 10^7^ total cells. 20 μL of FcR Blocking Reagent and CD133 MicroBeads were added per 10^7^ total cells, respectively. After mixing well and incubation at 2-8 °C for 15 min, cells were washed and resuspended up to10^7^ cells in 500 μL of buffer. The cell suspension was finally applied onto a MACS Column, and the unlabeled cells (CD133^−^) and magnetically labeled cells (CD133^+^) were collected repectively. Thereafter, the sorted CD133^+^ cells were seeded in ultra-low attachment 6-well plates (Corning Inc., NY, USA) for amplification culture with stem cell-conditioned medium.

### Flow cytometry analysis

The sorted CD133^+^ cells, CD133^−^ cells and unsorted parental NCI-H446 cells were washed with PBS, and were adjusted to the single cell suspension at a density of 1 × 10^5^ cells/mL, respectively. Cells were incubated with PE-conjugated anti-human CD133 antibody (Biolegend, San Diego, CA, United States) for 30 min at 4 °C in the dark, and mouse IgG2b-PE was used as an isotype control. Finally, The cell suspension was applied onto a flow cytometry analysis of the percentage of CD133^+^ cells.

### Tumor sphere formation assay

The self-renewal capacity of cells was evaluated using suspension culture in ultra-low attachment 6-well plates (Corning Inc., NY, USA) with stem cell-conditioned medium [20]. Single cell suspensions were prepared with stem cell-conditioned medium and were loaded into ultra-low attachment 6-well plates (2 × 10^3^cells/ml). After culture for 6 days, the number of tumor spheres formed were counted and pictured under a phase-contrast microscope (Nikon Eclipse TE2000-S). The sphere forming rate was calculated as the total number of tumor spheres formed/the total number of cells inoculated × 100 %. For drug-intervention experiment, different concentrations of FTVF were added to the medium prior to cells were inoculated. For secondary sphere formation assay, tumor spheres derived from CD133^+^ NCI-H446 cells were digested and prepared into single cell suspensions. After that, cells were seeded into ultra-low attachment 6-well plates at a density of 1 × 10^3^cells/mL, and no drugs was added in the procedure of secondary sphere formation assay.

The article "A candidate Chinese medicine preparation-Fructus Viticis Total Flavonoids inhibits stem-like characteristics of lung cancer stem-like cells" was retracted in 2022. Reasons: manipulated images; duplicated images; signs of a paper mill.

### MTT assay

Parental NCI-H446 cells and CD133^+^ SFCs were seeded at a density of 5 × 10^3^ cells/well in a 96-well plate pre-coated with 0.6 % agarose, respectively. The procedure for MTT assay and the calculation of relative cell proliferation inhibition rate have been previously described [19]. The IC50 value was calculated using the Prism software (GraphPad Software, San Diego, CA).

### In vitro cell migration and invasion assays

The migration and invasion assays were performed using 24-well uncoated or Matrigel (BD Biosciences, United States) coated Transwell chambers with 8.0-μm pore polycarbonate membranes (Corning Coster, Cambridge, MA, USA) as previously described [21]. Briefly, 600 μL DMEM with 10 % FBS was added to the 24-well culture plate (lower chambers). Then the Transwell chambers were inserted into the 24-well plate, and cells were resuspended in a serum and growth factor-free DMEM and loaded into chambers (1 × 10^4^ cells/100 μl). Following incubation at 37 °C, cells that migrated or invaded to the lower surface of the membrane were fixed and stained with hematoxylin-eosin or Wright-Giemsa. Finally, the stained cells were digitally imaged and counted under an optical microscope (OLYMPUS IX51, Japan). For drug-intervention experiment, cells were pretreated with different concentrations of FTVF for 24 h prior to the transwell chamber assay.

### Western blot analysis

Western blot procedures were performed as previously described [22]. The following primary antibodies were used: Mouse monoclonal antibodies anti-CD44, ALDH1, Bmi1, Nanog, Oct4, Twist, Snail, p-Akt (Ser473) and Akt. β-actin was used as an internal control. Signals were detected using Enhanced chemiluminescence Kit (Amersham Pharmacia Biotech Inc., Piscataway, NJ, USA).

### Nude mice tumorigenicity assay

The SPF male Balb/c-nu mice were obtained from the Hunan Slac Jingda Laboratory Animal Co., Ltd. (Yueyang, Hunan). All animal studies in this study were performed according to the experimental animal breeding and use guide of Hunan Laboratory Animal Management Committee after approved by the Ethical Committee of Hunan Normal University. 18 SPF male Balb/c-nu mice were randomly devided into three groups (6/group). CD133^+^ cells and parental cells in PBS were mixed 1:1 with Matrigel (BD Biosciences, San Jose, CA) and were injected subcutaneously into the flanks of the animals, respectively. The numbers of cells inoculated in three groups were 1 × 10^2^, 1 × 10^3^ and 1 × 10^4^/mouse for CD133^+^ SFCs, and 1 × 10^4^, 1 × 10^5^ and 1 × 10^6^/mouse for parental cells, respectively. The animals were maintained in accordance with standard guidelines for about 2 months for tumor appearance. The size of tumor nodules were measured using an caliper, and the volume was calculated using V (mm^3^) = L (the longest diameter) × W (the shortest diameter)^2^ × 0.5. At the end of experiment, the tumors were excised, weighed and divided into pieces to be fixed in neutral buffered formalin and embedded in paraffin and sectioned for a routine histological evaluation using hematoxylin and eosin (H&E) staining or for immunohistochemical analysis of CD44 and CD133.

The article "A candidate Chinese medicine preparation-Fructus Viticis Total Flavonoids inhibits stem-like characteristics of lung cancer stem-like cells" was retracted in 2022. Reasons: manipulated images; duplicated images; signs of a paper mill.

### Immunohistochemical examination

The xenografted tumor tissuses were fixed in 10 % formalin, embedded in paraffin and sectioned for immunohistochemical analysis. For immunohistochemical staining, the deparaffinized sections were incubated with 3.3 % H_2_O_2_ for 10 min to block endogenous peroxidase activity. The sections were then blocked with Tris Buffered Saline (TBS) containing 5 % normal goat serum for 30 min. After incubated with diluted corresponding primary antibodies (1:200 for mouse anti-CD133 antibody and 1:250 for mouse anti-CD44 antibody) and a secondary antibody, the signals were detected using an EnVision system (Dako, Carpinteria, CA, USA) and counterstained with hematoxylin .

### Statistics analysis

Results are shown as mean ± SD. Analysis of variance was performed with SPSS 15.0 software for Windows using one-way ANOVA and pair-wise comparison with *t* test. P < 0.05 was considered statistically significant.

## Results

### Magnetic separation of CD133^+^ cells from NCI-H446 cell line

NCI-H446 cells grew anchorage-dependently in DMEM supplemented with 10 % fetal bovine serum. After sorted by CD133 microbeads separation system, the percentages of CD133 expressing cells in unsorted parental cells, CD133^+^ and CD133^−^ subpopulation cells were examined by flow cytometry analysis. Results showed that the percentages of CD133 expressing cells were 91.85 ± 2.17 %, 0.03 ± 0.01 % and 1.71 ± 0.29 % in CD133^+^, CD133^−^ subpopulation and parental cells respectively (Fig. 1). The sorted CD133^+^ cells derived from NCI-H446 cell line were further cultured for amplification in stem cell-conditioned medium. And the generated CD133^+^ SFCs were used for the following experiment.

**Fig. 1:** CD133 expression of CD133^+^, CD133^−^ subpopulation cells and parental NCI-H446 cells. **a**, control; **b**, parental NCI-H446 cells; **c**, CD133^+^ subpopulation cells; **d**, CD133^−^ subpopulation cells; **e**, CD133 expression in the above four cells described by histogram. ^*^ *P* < 0.05 *vs* control, ^#^ *P* < 0.05 *vs* parental NCI-H446 cells

The article "A candidate Chinese medicine preparation-Fructus Viticis Total Flavonoids inhibits stem-like characteristics of lung cancer stem-like cells" was retracted in 2022. Reasons: manipulated images; duplicated images; signs of a paper mill.

### CD133^+^ SFCs from NCI-H446 cell line exhibited lung cancer stem cell characteristics

Figure 2a shows that sphere-forming rate of CD133^+^ SFCs was much higher than that of parental cells. Moreover, Fig. 2b shows that single cells dissociated from CD133^+^ SFCs could form secondary tumor spheres continuously. These results suggested that CD133^+^ SFCs possessed stronger self-renewal capacity. In line with these findings, it was shown by western blotting that the expression levels of self-renewal related transcription factors (Bmi1, Nanog and Oct4) and stem cell markers (CD44 and ALDH1) in CD133^+^ SFCs were much higher than that of parental cells (Fig. 2c).

**Fig. 2:** CD133^+^ SFCs from NCI-H446 cell line exhibited higher self-renewal capacity compared to that of parental cells. **a**, The sphere-forming rate of **CD133** ^**+**^ SFCs and parental cells (PC). **b**, Tumor sphere formation by single cell dissociated from **CD133** ^**+**^ SFCs derived from SCLC NCI-H446 cell line (200 × magnification). **c**, The expression levels of self-renewal related transcription factors (Bmi1, Nanog and Oct4) and stem cell markers were compared between **CD133** ^**+**^ SFCs and parental NCI-H446 cells at 48 h. **d**, In vitro invasion capacity were compared between **CD133** ^**+**^ SFCs and parental NCI-H446 cells (400 × magnification). **e**, The expression levels of invasion related transcription factors (Twist1 and Snail1) were compared between **CD133** ^**+**^ SFCs and parental NCI-H446 cells at 48 h

Considering that CSCs might play a vital role in the early cancer metastasis, we next seek to examine the invasion capacity of CD133^+^ SFCs and parental cells. Results showed that CD133^+^ SFCs exhibited a higher invasion capacity in vitro than parental cells. And western blot results also showed that compared to parental cells, CD133^+^ SFCs expressed a higher level of EMT related transcription factors Twist1 and Snail1 (Fig. 2d and e).

Furthermore, the *in vivo* tumorigenicity experiment results showed that 1 × 10^3^ CD133^+^ SFCs cells could initiated tumor formation 18 days after inoculated Balb/c-nu mice, as compared to 31 days of tumorigenic latent period for 1 × 10^5^ parental cells (Table 1, Fig. 3a). Meanwhile, staining results revealed that the transplanted tumors derived from CD133^+^ SFCs and parent cells exhibited the similar histological morphology (Fig. 3b). These results indicated that CD133^+^ SFCs showed higher tumorigeic potential than parent cells. And the immunohistochemical results also showed that the frequency of CD133 and CD44 expressing cells in tumor tissues derived from CD133^+^ SFCs were significantly higher than that derived from parental cells (Fig. 3c). These findings fully supported our hypothesis that the enrichment of LCSLCs contributed to the high tumorigeic potential of CD133^+^ SFCs. Taken together, all the above findings strongly suggested that CD133^+^ SFCs possessed CSCs characteristics, and could be defined as LCSLCs.

The article "A candidate Chinese medicine preparation-Fructus Viticis Total Flavonoids inhibits stem-like characteristics of lung cancer stem-like cells" was retracted in 2022. Reasons: manipulated images; duplicated images; signs of a paper mill.

**Table 1:** Comparison of tumor formation ability of CD133^+^ SFCs and parental NCI-H446 cells in Balb/c-nu mice (*n* = 6)

Cell type	Cells inoculated (n)	Tumor incidence(n/6)	Latency(d)
PCs	1 × 10^4^	0/6	–
	1 × 10^5^	3/6	31
	1 × 10^6^	6/6	23
CD133^+^ SFCs	1 × 10^2^	0/6	–
	1 × 10^3^	4/6	18
	1 × 10^4^	6/6	11

*PCs* parental NCI-H446 cells, *CD133* ^*+*^ *SFCs* CD133^+^ tumor sphere forming cells derived from NCI-H446 cell line

**Fig. 3:** CD133^+^ SFCs from NCI-H446 cell line exhibited higher *in vivo* tumorigeic capacity compared to that of parental cells. **a**, *In vivo* tumorigeic capacity was compared between SFCs and parental NCI-H446 cells. Up: Balb/c-nu mice were inoculated subcutaneously with 1.0 × 10^5^ parental cells in the left fore leg, and no xenograft was observed 4 weeks after inoculation. Down: Balb/c-nu mice were inoculated subcutaneously with 1.0 × 10^3^ SFCs in the right fore leg, and xenograft formed 4 weeks after inoculation. **b**, The transplanted tumors derived from SFCs and parental cells exhibited the similar histological morphology(HE staining) (100 × magnification). **c**, The expression levels of stem cell markers (CD133 and CD44) were compared between xenografts formed by SFCs and parental NCI-H446 cells (100 × magnification)

### FVTF inhibits self-renewal of LCSLCs

Self-renewal property is the key feature of CSCs, which enables CSCs to initiate and maintain tumors continiously. Thus exploring new chemotherapy drugs that can target the self renewal pathway of CSCs would be extremely important for cancer therapy. Results in this study showed that FVTF (0.1, 1, 3, 10, 30 μg/mL) could preferentially inhibit the proliferation of LCSLCs in a concentration-dependent manner, and the IC_50_ is 0.7 μg/mL, as compared to an IC_50_ of 3.7 μg/mL for parental cells (Fig. 4a). Moreover, the tumor sphere formation assays results also demonstrated that FVTF (0.5, 1.0, 2.0 μg/mL) could both significantly decrease the primary and secondary tumor sphere forming rates of LCSLCs (Fig. 4b and c). These findings indicated that FVTF could suppress the self-renewal capacity of LCSLCs. In accordance with the above findings, the results of western blot analysis also revealed that FVTF (0.5、1.0、2.0 μg/mL) decreased expression level of the self-renewal related transcription factors Bmi1, Nanog and Oct4 in a concentration-dependent manner (Fig. 4d).

The article "A candidate Chinese medicine preparation-Fructus Viticis Total Flavonoids inhibits stem-like characteristics of lung cancer stem-like cells" was retracted in 2022. Reasons: manipulated images; duplicated images; signs of a paper mill.

**Fig. 4:** FVTF inhibits self-renewal of LCSLCs. **a**, FVTF selectively inhibited the proliferation of LCSLCs in a concentration-dependent manner. **b** and **c**, FVTF significantly decrease the primary and secondary tumor sphere forming rates of LCSLCs. **d**, FVTF decreased expression level of the self-renewal related transcription factors Bmi1, Nanog and Oct4 in a concentration-dependent manner at 48 h. **e**, FVTF decreased the expression of stem cell markers CD 133 of LCSLCs in a concentration-dependent manner as analyzed by Flow cytometry analysis at 48 h. ISC: Isotype control, SFC: CD133^+^ sphere forming cells derived from NCI-H446 cells; F, FVTF decreased the expression of stem cell markers CD 44 and ALDH1 of LCSLCs in a concentration-dependent manner as analyzed by western blotting at 48 h

### FVTF decreases stem cell markers expression of LCSLCs

In order to investigate the effects of FVTF on stem cell markers expression of LCSLCs, we examined the expression level of CD133, CD44 and ALDH using Flow cytometry or western blot analysis. As shown in Fig. 4e and f, FVTF decreased stem cell markers expression of LCSLCs CD133, CD44 and ALDH1 in a concentration-dependent manner.

### FVTF inhibits migration and invasion of LCSLCs in vitro

Furthermore, we are tempted to examine the effects of FVTF on migration and invasion capacity of LCSLCs in vitro. Transwell results showed that FVTF (0.5, 1.0, 2.0 μg/mL) inhibited migration and invasion of LCSLCs in vitro in a dose-dependent manner (Fig. 5a and b). In line with these findings, It was found that the invasion related transcription factors Twist1 and Snail1 of LCSLCs were significantly down-regulated after treatment with FVTF of different concentrations (Fig. 5c).

**Fig. 5:** FVTF inhibited migration and invasion of LCSLCs in vitro. **a** and **b**, FVTF (0.5, 1.0, 2.0 μg/mL) inhibited migration and invasion of LCSLCs in vitro in a dose-dependent manner (200 × magnification). **c**, FVTF decreased expression levels of invasion related transcription factors Twist1 and Snail1 of LCSLCs in a concentration-dependent manner

### FVTF inhibits LCSLCs characteristics through down-regulation of p-Akt

It has been reported that PI3K-Akt pathway could promote self-renewal capacity of Hematopoietic stem cells (HSCs) through regulating polycomb group protein including Bmi1. Consequently, we are tempted to examine the phosphorylation level of AKT in LCSLCs. Western blot analysis results showed that activation of AKT was highly elevated in LCSLCs compared to that in parental cells (Fig. 6a). And FVTF (0.5, 1.0, 2.0 μg/mL) treatment could significantly decrease the phosphorylation level of Akt in LCSLCs (Fig. 6b). Futhermore, a PI3K specific inhibitor LY294002 was used in the following study. As shown in Fig. 6c, LY294002 of different concentrations could efficiently decrease the p-Akt level of LCSLCs derived from NCI-H446 cells. We also found that down-regulated expression of p-Akt by LY294002 significantly inhibited self-renewal capacity of LCSLCs (Fig. 6d). Moreover, results showed that LY294002 (5.0 μM) could efficiently decreased FVTF(1.0 μg/mL) inhibited sphere forming rate (Fig. 6e) and the invasion cell rate (Fig. 6f) of LCSLCs to a lower level, accompanied by further decreased expressions of self renewal and invasion related transcription factors of LCSLCs (Fig. 6g and h). In summary, these findings indicated that the constitutively activation of Akt was involved in maintaining self-renewal of LCSLCs, and decreased phosphorylation level of Akt contributed to the FVTF inhibited stem cell characteristics of LCSLCs.

The article "A candidate Chinese medicine preparation-Fructus Viticis Total Flavonoids inhibits stem-like characteristics of lung cancer stem-like cells" was retracted in 2022. Reasons: manipulated images; duplicated images; signs of a paper mill.

**Fig. 6:** FVTF inhibits LCSLCs characteristics through down-regulation of p-Akt. **a**, The expression levels of phosphorylated AKT were compared between SFCs and parental NCI-H446 cells. **b**, FVTF decreased phosphorylation levels of Akt in LCSLCs in a concentration-dependent manner. **c**, LY294002 down-regulated phosphorylation levels of Akt in LCSLCs in a concentration-dependent manner. **d**, LY294002 significantly decreased the tumor sphere forming rate of LCSLCs. **e**, LY294002 significantly enhanced the inhibition effects of FVTF on tumor sphere formation capacity of LCSLCs. **f**, LY294002 significantly enhanced the inhibition effects of FVTF on cell invasion capacity of LCSLCs. **g**, LY294002 significantly enhanced the down-regulation of self-renewal related transcriptional factors by FVTF in LCSLCs. **h**, LY294002 significantly enhanced the down-regulation of invasion related transcriptional factors by FVTF in LCSLCs

## Discussion

Despite all kinds of efforts exploited to combat lung cancer, this disease remains the most frequent cause of cancer-related deaths in China. It is now generally accepted that LCSLCs were the determining tumorigenic cells responsible for lung cancer initiation, development, metastasis and relapse after chemotherapy. Therefore, targeted eradication of LCSLCs is extremely vital for improving the prognosis or even recovery of lung cancer.

In the present study, we isolated, enriched and obtained the CD133^+^ SFCs from human lung cancer NCI-H446 cells, by CD133^+^ magnetic separation and stem cell-conditioned medium suspension culture method. The following results confirmed that this subpopulation of cells exhibited higher in vitro self renewal, invasion and tumorigenicity capacity over parental cells, accompanied by an upregulated expression level of stem cell markers, self-renewal and invasion related transcription factors. Collectively, these SFCs exerted stem-like cell characteristics and were defined as LCSLCs.

The article "A candidate Chinese medicine preparation-Fructus Viticis Total Flavonoids inhibits stem-like characteristics of lung cancer stem-like cells" was retracted in 2022. Reasons: manipulated images; duplicated images; signs of a paper mill.

Increasing new emerging data have reported that transcription factors Bmi1, Nanog and Oct4 have been implicated in regulating self-renewal and multi-directional differentiation potential of CSCs and adult stem cells. Park IK et al. has reported that Bmi1, a member of the polycomb group proteins, is essential for maintenance of adult self-renewing haematopoietic stem cells [23]. Another study by Abdouh M et al. also revealed that PcG proteins are involved in Glioblastoma multiforme (GBM) tumor growth and required to sustain cancer initiating stem cell renewal [24]. Nanog and Oct4 are the core transcription factors that maintaining the self-renewal and pluripotency of embryonic stem cells [25–28]. It has been reported that coexpression of Oct4 and Nanog promotes metastasis of lung adenocarcinoma by inducing cancer stem cell-like properties and epithelial-mesenchymal transdifferentiation [29]. In this study, we found that Bmi1, Nanog and Oct4 were highly expressed in SFCs derived from NCI-H446 cells compared to that in parental cells, as confirmed by western blot analysis. It indicated that the SFCs possessed self renewal and pluripotency properties.

It is generally accepted that most cancer related-deaths are attributed to the local invasion and distal migration, but not the primary tumor itself [30, 31]. CSCs were considered to play a pivotal role in the early metastasis of many kinds of human malignant tumors including lung cancer. In our study, it was demonstrated by Transwell assays that SFCs derived from NCI-H446 cells exhibted higher invasion capacity in vitro than parental cells. These results revealed that SFCs possessed high invasion and metastatic potential. The invasion related protein Snail was one member of the zinc-finger transcription factor Snail superfamily. It has been reported that Snail can directly or indirectly mediated epithelial-mesenchymal transition (EMT) which results in tumor cell invasion and metastases. In clinical practice, overexpression of Snail is associated with poor prognosis and increased invasioness in several type of cancer patients [32–34]. Twist1, which belonged to the basic Helix-Loop-Helix (bHLH) transcription factor family, is a highly evolutionally conserved transcription factor firstly found in *Drosophila* and initially involved in embryo development by contributing to cell migration. A study from Mikheeva et al. has reported that TWIST1 promotes invasion through activation of mesenchymal molecular and cellular changes in human glioblastoma [35]. Li et al. has revealed that Twist1 depletion completely blocked the mesenchymal transformation induced by Adriamycin [36]. Our previous study also found that Twist signaling involved in maintaining self-renewal and invasion properties of liver cancer stem cells. In this study, we showed that the EMT-related transcription factors Snail and Twist1 were highly expressed in SFCs as compared to that in parental cells. Although no gene expression regulation measures were further taken, we have reasons to speculate that the high invasion capacity of SFCs may be related to its high expression level of Snail1 and Twist.

The article "A candidate Chinese medicine preparation-Fructus Viticis Total Flavonoids inhibits stem-like characteristics of lung cancer stem-like cells" was retracted in 2022. Reasons: manipulated images; duplicated images; signs of a paper mill.

Since increasing studies have proved that there exists a plenty of active compounds with anti-cancer properties in some phytomedicines, extracting and isolating anti-cancer agents from naturally-occurring plants becomes one of the main approaches for new anti-tumor drugs discovery. In the present study, we demonstrated that the candidate Chinese medicine preparation FVTF could relative selectively inhibit the proliferation and self-renewal, and suppress migration and invasion of LCSLCs in vitro. In agreement with above findings, we also found that FVTF down-regulated the protein expression of stem cell markers (CD133, CD44 and ALDH1), self-renewal associated transcription factors (Bmi1, Nanog and OCT4) and invasion associated transcription factors (Twist1 and Snail1) in a dose-dependent manner. Furthermore, we demonstrated that the inhibitory effects of FVTF on LCSLCs characteristics appeared to be mediated through down-regulating expression of p-Akt.

Akt, also known as protein kinase B(PKB), is a multifunctional serine-theonine protein kinase involved in a variety of biological functions in cells. A recent study has reported that Akt activation in Hair follicle stem cells (HF-SCs) results in increased tumor development and malignant transformation [37]. Chen et al. showed that Akt could phosphorylate Oct4 at threonine 228 to accelerate its degradation. And Akt mediated phosphorylation of special AT-rich sequences binding protein 1 (SATB1) played a key role in inhibiting Nanog expression [38]. Another study by Wang et al. found that AKT/β-catenin/Snail signaling pathway is mechanistically involved in acquisition of cancer stem cell-like properties and EMT features in cisplatin-resistant A549 cells [39]. In this study, we also showed that the constitutively activation of Akt was involved in maintaining self-renewal of LCSLCs. And the use of FVTF or LY294002 could significantly decrease the phosphorylation level of Akt in LCSLCs. Interestingly, we also found that LY294002 could act alone or synergize with FVTF to suppress the characteristics of LCSLCs. Therefore, it is reasonable to speculate that FVTF may inhibited the phosphorylation of Akt by a pathway different from the way that LY294002 acted in.

The article "A candidate Chinese medicine preparation-Fructus Viticis Total Flavonoids inhibits stem-like characteristics of lung cancer stem-like cells" was retracted in 2022. Reasons: manipulated images; duplicated images; signs of a paper mill.

Taken together, our results have demonstrated that FVTF can inhibit characteristics of LCSLCs derived from NCI-H446 cell line. And the mechanisms is probably associated with down-regulating expression of p-Akt in LCSLCs, which lead to downregulation of the expressions of stem cell markers, self-renewal associated transcription factors and invasion associated transcription factors. However, based on the limitation of conducting these experiments in a single cell line derived LCSLCs, future efforts would be made toward confirming the therapeutic effects of FVTF in more cell lines as well as in animal model.

## Conclusions

FVTF inhibits characteristics of lung cancer stem-like cells through down-regulating expression of p-Akt.

## Abbreviations

ALDH1: Aldehyde dehydrogenase 1
CSCs: Cancer stem cells
FVTF: Fructus viticis total flavonoids
LCSCs: Lung cancer stem cells
LCSLCs: Lung cancer stem-like cells
NSCLC: Non-small cell lung cancer
SCLC: Small cell lung cancer
SFCs: Sphere-forming cells.
